# Development, Biological Characterization, and Immunological Evaluation of Virosome Vaccine against Newcastle Disease in Pakistan

**DOI:** 10.1155/2021/8879277

**Published:** 2021-01-29

**Authors:** Muhammad Hidayat Rasool, Asif Mehmood, Muhammad Saqalein, Muhammad Atif Nisar, Ahmad Almatroudi, Mohsin Khurshid

**Affiliations:** ^1^Department of Microbiology, Government College University Faisalabad, Pakistan; ^2^Department of Medical Laboratories, College of Applied Medical Sciences, Qassim University, Buraydah, Saudi Arabia

## Abstract

Newcastle disease (ND) is a highly fatal, infectious, viral disease, and despite immunization with live and inactivated vaccines, the disease is still endemic, causing heavy morbidity and mortality leading to huge economic losses to the poultry industry in Pakistan. Therefore, the present study was aimed for the first time in the country at using novel virosomal technology to develop the ND vaccine using an indigenous highly virulent strain of the virus. ND virosome was prepared using Triton X-100, and SM2 Bio-Beads were used to remove the detergent and reconstitute the viral membrane into virosome. Confirmation was done by transmission electron microscopy and protein analysis by SDS-PAGE. *In vitro* cell adhesion property was observed by incorporating green fluorescent protein (GFP), producing plasmid into virosome and *in vitro* cell culture assay. Sterility, safety, and stability of the vaccine were tested before *in vivo* evaluation of immunogenicity and challenge protection study in commercial broiler. The virosome vaccine was administered (30 *μ*g/bird) at days 7 and 14 through the intranasal route in comparison with commercially available live and inactivated ND vaccines. Results revealed significantly high (*p* < 0.05) and clinically protective hemagglutination inhibition (HI) antibody titers at 7, 14, 21, and 28 days postimmunization with the virosome vaccine in comparison to the negative control. The GMTs were comparable to live and inactivated vaccines with nonsignificant (*p* > 0.05) differences throughout the experiment. Antibody levels increased in all vaccinated groups gradually from the 7^th^ day and were maximum at 28^th^-day postvaccination. In the virosome-administered group, GMT was 83.18 and 77.62 at 21^st^ and 28^th^-days postvaccination, respectively. Challenge revealed 100%, 90%, and 80% protection in virosome, live, and inactivated vaccinated groups, respectively. Under given experimental conditions, we can conclude that ND virosome vaccine prepared from the indigenous virus was found to be safe and immunogenic.

## 1. Introduction

The poultry industry is one of the leading industries and a source of income for more than 21 million people, contributing 23.8% of total meat production in Pakistan. However, it is facing severe economic losses due to the number of infectious diseases such as Newcastle disease (ND). The outbreaks of ND have been reported from all continents of the world including Africa, Asia, Europe, Australia, and South and Central America [1, 2]. This is one of the deadliest infections of poultry and results in heavy mortality in all ages of chicken [3, 4].

According to the International Committee on Taxonomy of Viruses (ICTV), Newcastle disease virus (NDV) belongs to the family Paramyxoviridae, subfamily Paramyxovirinae, and genus Avulavirus. It is the only member of Avian Paramyxovirus Type 1 (APMV-1) and affects all the domestic and wild birds [5]. NDV is an enveloped virus with an RNA genome, which is a negative sense, single-stranded, nonsegmented, and has about 15 kb length. The genome is translated into six major structural proteins which are encoded from 5′ to 3′ direction. These include a large RNA-dependent RNA polymerase (L), Hemagglutinin-Neuraminidase (HN), Fusion protein (F), Matrix protein (M), Phosphoprotein (P), and Nucleoprotein (NP) [6, 7].

Class II genotype III NDV has been recovered from Asia, South America, Africa, and Europe. These viral strains are most used in the formation of live and inactivated vaccines. The viruses of this genotype have been recognized as velogenic NDVs, which increase their economic significance in poultry. Many strains identified in poultry arise due to the administration of live vaccines, and they used to circulate in poultry products world widely [8, 9]. Class II genotype IV isolates have been reported in poultry from Africa, Russia, and Europe and in pigeons from Asia. These viruses are pathotyped as virulent NDV and include a well-known strain Herts/33 [10]. Class II genotype V NDVs can be either mesogenic or virulent, which is evident from gene sequencing and pathotyping.

Although virulent NDV has been isolated from certain areas of Pakistan, it is of utmost importance to identify and characterize virulent strains from all over the country. These studies have a potential role in the emergence of novel virulent NDV genotypes, which is being reported recently. In Asia NDV, genotype VII is still prevalent in domestic poultry, and they were found identical to the strains isolated back in the 1990s. Homologous isolates can be used for immunization purposes, and the vaccination programs can be optimized according to environmental circumstances [11].

Newcastle disease virus is considered as endemic throughout the year in Pakistan. However, extensive vaccination programs have been initiated in the past decades to mainly protect commercial poultry farms, and to some extent, the rural poultry as well which has resulted in a low number of NDV outbreaks in Pakistan. At present, live attenuated vaccines are in use which includes La Sota or Mukteswar strain followed by the administration of Mukteswar or Komarov strain. These strains impart immunity to day-old chicks but are unable to completely control the disease as sporadic outbreaks do occur. Such failures have put many question marks on the efficacy of these vaccines. Vaccination failure has many reasons like an incompatibility between the field and vaccinal strains, poor vaccination techniques, and the formation of new genotypes under high immune pressure [12].

To overcome this problem, a novel approach like the use of virosome (s) has to be explored in Pakistan, which involves the use of surface components of virulent viral strains. Virosome consists of nonreplicating virus particles, which are reconstituted viral membranes having surface glycoproteins. This technique has proven successful for the preparation of a vaccine against other viruses like the Sendai virus, Respiratory Syncytial Virus (RSV), and Influenza virus. Moreover, virosomes can be easily combined with lipophilic adjuvants, such as viral protein antigens mixed with lipophilic TLR-ligands [13].

The virosomal vaccines are alike the live attenuated vaccines as these induce both humoral as well as cell-mediated immunity with the added advantage of nonreversion as the nucleocapsid has already been removed during the synthesis process [13, 14]. Moreover, the inactivated vaccines fail to induce cell-mediated immunity, but virosomal vaccines are processed by both MHC-I and MHC-II pathways, hence, activating the humoral as well as cellular immunity. In humans, these vaccines have been reported to be equally effective in individuals with autoimmune disorders and even in patients of human immunodeficiency virus (HIV) infection [15–17].

The increasing number of outbreaks and high prevalence of ND exhibit that although live and inactivated ND vaccines are used worldwide but these vaccination strategies are unable to control the disease. However, these vaccines are manufactured using embryonated egg-based technologies which nevertheless have many disadvantages, e.g., low yields, laborious, potential biohazard, and often have contaminants [18]. Virosomes are virus-like particles (VLPs), a group of novel putative vaccines constituted from glycoproteins of the virus, maintaining similarity and spatial antigenicity to live virus and without the risk of viral replication [19].

Therefore, the present study was conducted for the first time in Pakistan to use novel virosome technology to develop, characterize, and evaluate ND vaccine using indigenous very virulent NDV.

## 2. Materials and Methods

### 2.1. Isolation and Identification of Virus from Field Outbreaks

Samples were obtained from different field outbreaks of ND in broiler flocks located in district Okara Punjab Pakistan. Trachea, spleen, lung tissues, cloacal, and tracheal swabs were collected aseptically [20], processed and filtrates were cultured in nine days old embryonated chicken eggs [21]. After 48 hours of incubation, allantoic fluids were harvested and filtered through 0.2 *μ*m syringe filters. Filtered allantoic fluids were subjected to microhemagglutination assay to observe the agglutination pattern and virus titration [22]. Each viral filtrate depicting hemagglutination activity was confirmed through HI assay using the known hyperimmune serum for confirmation of NDV [23].

### 2.2. Purification of Virus

The virus was purified from allantoic fluids by sucrose gradient ultracentrifugation technique [21]. Briefly, 20%, 30%, and 50% (*w*/*v*) sucrose solutions were prepared in deionized double distilled water and filtered by using 0.2 *μ*m filter paper (Whatman® membrane, Sigma Aldrich, USA). The sucrose gradient was established by adding 50% (5 ml), 30% (5 ml), and 20% (5 ml) sucrose in sterile centrifuge tubes. Finally, sterilized and positively confirmed embryonic allantoic fluid (5 ml) through HI assay was layered over sucrose layers. The centrifuge tubes were balanced and ultracentrifuged at 120,000 × g for 120 minutes at 4°C (Type 90 Ti rotor, Optima L-100XP, Beckman Coulter, USA). Then, tubes were ethanol sterilized, and a clear middle layer (band) containing purified virus was collected and transferred to sterile 15 ml falcon tubes (Corning®, Sigma-Aldrich, USA), using sterile 5 ml syringes (Becton Dickinson, USA). To remove any residual impurity, the purified virus was again filtered through a 0.2 *μ*m syringe filter (Whatman® membrane, Sigma Aldrich, USA). Finally, the purified virus was aliquoted into 1.5 ml microcentrifuge tubes (Corning®, Sigma-Aldrich, USA) and stored at -70°C (Innova® U725, New Brunswick laboratory freezer, Eppendorf, Germany).

### 2.3. Assessment of Pathogenicity

*In vivo* pathogenicity of purified NDV was determined by calculating the Intra Cerebral Pathogenicity Index (ICPI) in chicks, Mean Death Time (MDT), and Embryo Lethal Dose_50_ (ELD_50_) in embryonated chicken eggs using standard protocols [23]. The ICPI value (mean score/bird) was calculated and interpreted as virulent strains 2 scores, whereas lentogenic (nonpathogenic) strains score near to 0 [24].

### 2.4. Amplification and Sequencing of Fusion Gene

Total genomic RNA from purified NDV was extracted using QIAamp viral RNA mini kit (Qiagen™, USA) as per manufacturer's recommendations [25]. Purified RNA was quantified spectrophotometrically (UV-1900 UV-Vis spectrophotometer, Shimadzu, Japan) and used for the synthesis of complementary DNA (cDNA). Commercially available SuperScript™ III reverse transcriptase kit (Thermo-Fisher™ Scientific, USA) was used for the generation of the first-strand cDNA. Finally, purified cDNA was stored at -70°C (Innova® U725, New Brunswick laboratory freezer, Eppendorf, Germany). The cDNA was used for the amplification of the viral fusion gene using the following specific primers chemically synthesized from Macrogen, Korea [26].

Forward oligomer TGGAGCCAAACCGCGCACCTGCGG

Reverse oligomer GGAGGATGTTGGCAGCAT

Amplicons were visualized in ethidium bromide-stained 1% agarose gel, and size was estimated using a 1 kb DNA ruler (New England Biolabs®, USA) [27]. PCR amplicons were purified using the QIAquick PCR purification kit (Qiagen™, USA), as per the guidelines of the manufacturer. Purified products were dispatched for di-deoxy Sanger's sequencing from Macrogen, Korea. Sequences obtained from Macrogen, Korea, were analyzed using different bioinformatics tools and online programs [28, 29]. Genetic and evolutionary relatedness of the fusion gene were analyzed, and a phylogenetic tree was constructed by the neighbor-joining method [29].

### 2.5. Protein Analysis and Mass Spectrometry

Viral proteins were analyzed by one-dimensional denaturing gel electrophoresis. The viral samples were processed and electrophoresed via vertical gel electrophoresis [27]. The NDV was identified based on the number and molecular weights of different bands of proteins. The protein band equivalent to fusion protein was excised out and subjected to in the gel digestion [30]. The eluted bands were subjected to mass spectrometry, and the size of the peptide was estimated [31]. Finally, the Mascot search engine (Matrix Science, USA) was used for peptide analysis and comparison to MSDB and Swiss-Prot databases.

### 2.6. Preparation and Confirmation of ND Virosomes

The ND virosomes were constructed using isolated and characterized local strain of NDV responsible for field outbreaks in district Okara region of Punjab Pakistan as described [14, 32]. Briefly, purified virus particles were dissolved in 1X PBS (phosphate-buffered saline, pH 7.2), and protein quantity was estimated by Bradford protein estimation assay (Bio-Rad, USA) [32, 33]. Then, 5 mg/ml viral suspension was mixed with detergent Triton X-100 (Sigma-Aldrich, USA), and the final concentration of detergent was maintained up to 2% (*v*/*v*). The mixture was placed on a rocking platform at room temperature for 60 minutes. The viral suspension was ultracentrifuged at 120,000 × g for 60 minutes at 4°C (Type 90 Ti rotor, Optima L-100XP, Beckman Coulter, USA). The supernatant was carefully transferred to a sterile tube, whereas the pellet was discarded as the viral nucleocapsid.

SM2 Bio-Beads (Bio-Rad, USA) was used to remove the detergent and reconstitute the viral membrane into virosome. Briefly, 150 mg SM2 Bio-Beads were inoculated into 2 ml viral supernatant and placed on a shaking incubator at 25°C for 120 minutes followed by the addition of 300 mg SM2 Bio-Beads and incubation at 4°C for 120 minutes. Finally, 600 mg of SM2 Bio-Beads was added, and the mixture was incubated overnight at 4°C. Later, reconstituted virosomes were carefully collected by a syringe and transferred to a sterile microcentrifuge tube. Protein contents of prepared virosomes were quantified by Bradford protein estimation assay. Quantified virosomes were aliquoted in 1.5 ml sterile microcentrifuge tubes and stored at -70°C (Innova® U725, New Brunswick laboratory freezer, Eppendorf, Germany).

The construction of a proper virosome was confirmed by transmission electron microscopy (TEM). Virosome samples were processed and visualized by JEM-1210 TEM (Jeol, USA) as described [14]. Moreover, protein contents of virosomes were analyzed by SDS-PAGE and compared with proteins of the whole NDV.

### 2.7. Biological Characterization of ND Virosomes

Fusion studies of prepared virosomes were done by incorporating green fluorescent protein (GFP) producing plasmid into the virosome and through *in vitro* cell culture assay. AcGFP1-C1 plasmid (Addgene, USA) was amplified in *Escherichia coli* DH5*α* cells and after extraction inoculated on Vero cells (*Cercopithecus aethiops* kidney epithelial cells, CCL-81™, ATCC®, USA) [34]. The plasmid was obtained from the Department of Biology, Lahore University of Management Sciences (LUMS), Pakistan, and the Vero cell line was provided by Quality Operations Laboratory, the University of Veterinary and Animal Sciences (UVAS) Lahore, Pakistan.

### 2.8. Preparation and Transformation of Competent E. coli DH5*α*

*Escherichia coli* DH5*α* is a genetically modified bacterium, capable to increase the copy number of plasmids. The competent cells were produced by chemical methods. The competent *E. coli* DH5*α* was transformed with AcGFP1-C1 plasmid, and kanamycin was used as a selection antibiotic. The transformed cells were cultured in kanamycin (50 *μ*g/ml) containing LB broth, and plasmids were extracted by alkaline lysis method using QIAprepspin Miniprep kit (Qiagen, Germany) [27].

### 2.9. Plasmid Incorporation in Virosome

The supernatant obtained from ultracentrifugation containing virus-detergent suspension was mixed with plasmid and placed at room temperature for 60 minutes. To remove detergent, the mixture was treated with SM2 Bio-Beads as mentioned earlier, and plasmid harboring virosome was reconstituted. Protein contents of virosomes were quantified by Bradford assay and stored at -70°C (Innova® U725, New Brunswick laboratory freezer, Eppendorf, Germany). The incorporation of the plasmid in the virosome was confirmed by nested polymerase chain reaction using the following primers synthesized from Macrogen, Korea [27].

Forward Primer (CMV-F)CGCAAATGGGCGGTAGGCGTG

Reverse Primer (SV40-pArev)CCTCTACAAATGTGGTATGG

### 2.10. Virosome-Cell Fusion Assay

Fusion studies were conducted to decipher the potential of the virosome to bind with animal cells, *in vitro*. Vero cells originated from monkey (*Cercopithecus aethiops*) kidney epithelium were cultured and maintained under standard cell culture conditions. The standard protocol was used for cell culturing and maintenance [35]. After cell attachment, the culture medium was replaced with 500 *μ*l serum-free RPMI-1640. Then, in one well plasmid containing virosomes was inoculated, whereas the second well was inoculated with plasmid-free virosomes, while the third well was left as a negative control. As positive control cells were inoculated with plasmid-lipofectamine (Thermo-Fisher™ Scientific, USA) mixture. To prepare the mixture, the plasmid was resuspended in lipofectamine with a ratio of 5 : 1 and incubated at room temperature for 60 minutes. After 1-hour incubation, the medium of each well was replaced with 1.5 ml RPMI 1640, supplemented with 5% HI-FBS. Then, cells were further incubated for 48 hours under standard culture condition. After 48 hours of incubations, coverslips were taken out and cells were examined under a camera-fitted fluorescent microscope (Optika®, Italy) and images were captured.

### 2.11. Development and Evaluation of Virosome Vaccine

The ND virosome after *in vitro* characterization and fusion studies in cell culture were evaluated as a vaccine. Sterility, safety, and stability of virosome-based vaccine were tested using standard protocols as per recommendations of the OIE safety manual before the *in vivo* evaluation of immunogenicity and challenge protection study in experimental broiler birds.

#### 2.11.1. Commercial Vaccines

In this study, the Newcastle disease vaccine (La Sota Live) (NDVL) manufactured by Veterinary Research Institute, Lahore, Punjab, Pakistan (VRI, Lahore), was used. Vaccine was composed of chicken embryo adapted La Sota strain of NDV with each dose containing at least EID_50_ = 10^6.5−7^. Each vial contained 200 doses (mixed with 2 L of sterile water before administration) in the form of a freeze-dried pellet. The recommended route is through eye drops or intranasal initially and later through drinking water. Whereas Medevac ND Emulsion manufactured by Medion Bandung Indonesia and marketed by Hilton Pharma Pakistan was used as killed vaccine and it contained Newcastle disease (ND) virus of La Sota strain. The virus was emulsified in mineral oil adjuvant. Each dose contained at least 50 PD_50_ ND virus, the dosage is 0.2 ml per young chicken or 0.5 ml per adult chicken given intramuscularly (through muscle) on thigh/breast or subcutaneously (under the skin) at the lower back of the neck.

#### 2.11.2. Experimental Design

One-hundred-day-old broiler chicks were purchased from a commercial hatchery and reared at the “Experimental Broiler Farm” Pattoki, Department of Poultry Science, University of Veterinary and Animal Sciences Lahore Pakistan. This experimental center had controlled temperature and humidity conditions with automated water and feed supply. The chicks were given standard poultry feed, and drinking water was provided *ad libitum*. The experiment was carried out under the regulations of the Institutional Animal Care, and all the guidelines were followed for the rearing of broiler chicks. Daily feed intake, morbidity, and mortality record were kept throughout the experiment. The chicks were divided into four equal groups (G1, G2, G3, and G4) having (*n* = 25) birds in each group. Group 1 was vaccinated with the virosome NDV vaccine (30 *μ*g/bird) at days 7 and 14 through the intranasal route. Group 2 was vaccinated with ND La Sota live vaccine (VRI, Lahore) as per manufacturer instructions on day 5 and day 12 through the intranasal route. Group 3 was inoculated with the 0.2 ml of killed vaccine (Medevac ND Emulsion) per chick at day 5 and day 12 via the intramuscular route. Group 4 was kept as negative control and inoculated with 100 *μ*L of PBS. A booster dose was given at day 14 of age [36].

#### 2.11.3. Immunogenicity of Vaccines

Blood samples were drawn before vaccination and at days 7, 14, 21, and 28 postimmunization from 10 birds at random in a group using EDTA coated vacutainers (Improv, China). Later on, sera were separated, heat-inactivated in a water bath at 56°C for 30 minutes, and kept in aliquots at -20°C until used for measuring antibody titers using HI test [36].

### 2.12. Challenge Protection Study

A challenge protection assay was performed to evaluate the efficacy of the virosome vaccine in comparison to commercially available ND vaccines. The ten randomly selected birds in each group were challenged with a local strain of Velogenic NDV (10^4^ EID_50_/chick) intramuscularly using 0.1 ml inoculum at 21 days postvaccination. Clinical signs of the disease (torticollis, muscle tremors, paralysis of legs and wings, etc.) were observed twice daily, and mortality was recorded up to 10 days of postchallenge. The protective efficacy was calculated by dividing the number of birds that survived the challenge by the total number of birds challenged as described [36].

### 2.13. Statistical Analysis

The immunization titers were statistically analyzed by calculating geometric mean titers (GMTs) and through one-way analysis of variance (ANOVA). The statistical differences in antibody titers among different vaccinated groups in comparison to negative control were further studied using the least significant difference (LSD) test at a confidence level of 95%. All the analyses were performed using SPSS version 13.0 for Windows [37].

## 3. Results

### 3.1. Isolation and Characterization of ND Virus

Indigenous ND virus was successfully isolated from field outbreaks of Newcastle disease in commercial broiler birds from in and around the Okara district of Punjab, Pakistan, from June 2017 to March 2018. All these outbreaks resulted in very high levels of mortality (up to 83% on average) in vaccinated flocks. Initially, spot agglutination test and then microhemagglutination (HA) assay was used for the identification and titration of NDV from harvested allantoic fluids followed by confirmation through HI assay using a known hyperimmune serum. The virus titer was found to be 256 HAU, which was used to calculate the 4 HAU. The inhibition of hemagglutination ability by specific antibodies confirmed the presence of ND virus. The ICPI score of isolated NDV was found as 2, representing the highest level of virulence of the virus. Moreover, the MDT score was less than 50 hours and 10^8.5^ ELD_50_/ml, which indicates that all the local isolates of NDV from filed outbreaks were highly virulent or velogenic.

### 3.2. Molecular Characterization

Genetic confirmation of NDV was done by amplification of the viral fusion gene. Amplicons were visualized on ethidium bromide-stained 1% agarose gel, and the mass of the product was estimated at approximately 800 bp using a DNA ladder (Figure 1). The protein-coding region of the sequence was submitted to GenBank with accession number MH607122 via BankIt, NCBI. Phylogenic analysis revealed that our virus was closely related (identity nearly 99%) to the UVAS-2015 strain (Accession No. MF437287, Lahore Pakistan origin) followed by the UVAS-2016 strain (Accession No. KX91187, Lahore Pakistan origin) and Tehran strain (Accession No. MG871466, Tehran Iran origin) (Figure 2).

In SDS-PAGE analysis, based on molecular mass, five different viral proteins were identified as viral hemagglutinin-neuraminidase (HN), fusion (F), nucleocapsid (NP), phospho (P), and matrix (M) proteins, respectively (Figure 3). For proteomic profiling of indigenous NDV strain, the protein band corresponding to fusion protein (approximately 55 to 60 kDa) was excised out from the gel and subjected to in-gel digestion. Afterward, the peptide mixture was analyzed by mass spectrometry. From Mascot search engine analysis and comparison to MSDB and Swiss-Prot databases, the mass of peptides was estimated as 58896.0 Da and identified as a viral fusion protein with Accession No. AAC28374.

### 3.3. Preparation and Characterization of Virosome

The constructed virosome was structurally like the wild type NDV. Electron micrographs represented circular to oval-shaped virosomes with the size ranging from 75 to 200 nm (Figure 4). Results of SDS-PAGE revealed that in comparison to five viral proteins identified in the whole virus, ND virosomes contained only two proteins, i.e., hemagglutinin-neuraminidase (HN) and fusion (F) (Figure 5). Both HN and F protein are membrane proteins present on viral envelop and are responsible for the adhesion of virion with host cell as well as immunogenicity.

### 3.4. In Vitro Fusion Studies of Virosomes

The AcGFP1-C1 plasmid containing virosomes were confirmed by amplification of plasmid using CMV-F and SV40-pArev primers. Virosomes were subjected to nested PCR, and amplicons of 900 bp were observed by agarose gel electrophoresis (Figure 6).

Confirmed AcGFP1-C1 plasmid containing virosomes were used for the transfection of Vero cells monolayer. After 48 hours of transfection, cells were visualized under bright field and fluorescent microscopic fields. Green color fluorescence was observed in the AcGFP1-C1 plasmid containing virosome transfected cells, whereas negative control (untransfected) cells did not produce any fluorescence (Figure 7). These results revealed the presence of intact viral envelop proteins (HN and Fusion) on ND virosomes and thus confirmed their fusion ability to animal cells *in vitro*.

### 3.5. Evaluation of Virosome Vaccine

Results showed that the virosome vaccine exhibited good seroconversion. The HI antibody titers were protective and the highest in G2 vaccinated with a live vaccine, followed by virosome (G1) and killed (G3) vaccines, respectively. The GMTs were very low and nonsignificant (*p* > 0.05) in all groups before vaccination, whereas a significant difference (*p* < 0.05) in GMTs was observed in all vaccinated groups from the negative control group (G4) throughout the experiment. The antibody titers were maximum in the virosome vaccine group (G1) with the highest GMTs as 83.18 and 77.62 at 21^st^ day and 28^th^-day postvaccination, respectively. Likewise, titers were also found maximum in the case of the live vaccine group (G2) with GMTs values as 89.13 and 77.62 at 21^st^ day and 28^th^-day postvaccination, respectively. A similar trend was also observed for the killed vaccine (G3) with nonsignificant (*p* > 0.05) differences in GMTs as compared to virosome and live ND vaccines. The comparative GMTs in different groups at different days postvaccination have been presented in (Tables 1 and 2).

### 3.6. Challenge Protection Assay

In challenge protection assay, the virosome vaccine showed 100% protection, whereas commercially available live vaccine (La Sota) and killed vaccines exhibited 90% and 80% protection, respectively. The percentage morbidity, percentage mortality, and protection percentage up to 10 days postchallenge have been shown in Table 3.

## 4. Discussion

Since 1926, the year NDV was reported for the 1^st^ time, about 9 genotypes have been identified depicting a diverse and continued evolution. The new genetic variants of NDV are being reported from different regions of the world with varying virulence highlighting that discrete genotypes of NDV are continuously evolving in distinct geographic areas of the world [31, 38]. Currently, along with strict biosecurity measures, many live and killed vaccines are being used on a mass scale throughout the world to control and prevent ND [39, 40]. Conventional strategies for vaccine development mainly focus on inactivated vaccines, recombinant protein vaccines, and modified live vaccines.

In the current study, highly virulent NDV was isolated from a field outbreak of the disease in vaccinated birds from district Okara, Pakistan. All these outbreaks resulted in very high levels of mortality (up to 83% on average) in vaccinated broiler flocks [6, 20, 41]. Many previous reports are suggesting the risk of substantial mortality even in vaccinated flocks [42]. The most important reason may be that vaccines can protect birds against clinical outcomes and mortality, but unable to block virus shedding among postvaccinated healthy birds, which are the main cause of disease spread [12, 43].

ND virus was cultivated in embryonated chicken eggs for propagation, and allantoic fluid was harvested. Initial screening was achieved by slide agglutination assay with known antiserum. Titer 1 : 32 to 1 : 256 HAU was obtained in the microhemagglutination test. The presence of NDV was confirmed through the HI assay. These findings are consistent with previous studies [3, 44]. The sucrose gradient ultracentrifugation was adopted for purification of the virion from the allantoic fluid as also reported in an earlier study [21].

The most appropriate method to characterize NDV is sequence analysis of fusion gene and protein profiling, an amplified product of the viral fusion gene was visualized on ethidium bromide-stained 1% agarose gel. The size of the band was approximately 800 bp estimated by the DNA ladder which is coherent with the previous studies [25, 34, 45, 46]. Our strain (Accession No. MH607122) displayed the highest identity (approximately 99%) with already known strains reported from Lahore, the UVAS-2015 strain (Accession No. MF437287) and UVAS-2016 strain (Accession No. KX91187) [1, 25, 47]. After Lahore strains, it displayed the highest levels of identity with the Tehran strain (Accession No. MG871466). According to phylogenetic analysis, our Okara strain revealed identity with different Asian (Iran, China, Japan, Malaysia, and Indonesia) and European (Ukraine and Netherland) strains, available on GenBank, NCBI, our findings also correlate with a recent report [25].

SDS-PAGE and Western blotting are rapid and appropriate methods to study the antigenic viral proteins [48]. Viral proteins were characterized by SDS-PAGE analysis, and a total of five different viral proteins were identified as hemagglutinin-neuraminidase, fusion, nucleocapsid, phospho, and matrix proteins. In SDS-PAGE gel, two distinct prominent signature protein bands corresponding to major glycoproteins; the hemagglutinin-neuraminidase and fusion protein, whereas a third band of the matrix proteins was observed which was similar to earlier reports [34, 36, 45]. Mass spectrophotometric analysis of protein band comparable to fusion protein was performed. Two distinct spectral peaks were observed in the spectrum of the fusion protein. According to MS database search engines, the selected band was identified as a viral fusion protein with 58896.0 Da and characterized as a viral fusion protein (Accession No. AAC28374) [14, 34, 36]. The results are comparable to data available on UniProt, TrEMBL, and Swiss-Prot database (https://www.uniprot.org/uniprot/O90339). The existence of fusion protein indicates the highly pathogenic nature of the virus [8, 49, 50].

According to ICPI results, the isolated virus belonged to a highly virulent strain with a maximum intracerebral pathogenicity index score of 2 [51–53]. Moreover, the MDT score was less than 50 hours and 10^8.5^ ELD_50/_ml, which confirmed that the NDV strain Okara/Pakistan/MH607122 isolated from the filed outbreak was highly virulent or velogenic [23].

Transmission electron micrographs represented circular to oval-shaped virosomes with the size ranging from 75 to 200 nm, and constituted virosome was structurally similar to the wild type of NDV which corroborates the previous findings [14, 34]. SDS-PAGE confirmed the presence of both HN and F membrane glycoproteins on viral envelop and are responsible for the adhesion of virion with host cells as well as immunogenicity, corresponding to the observations of previous studies [14, 34].

The fusion of the virosome to host cells is important to induce the activation of the immune system [54]. Fusogenic properties of virosomes can be studied *in vitro* using animal cell culture. In the present study, green fluorescent protein-encoding plasmid (AcGFP1-C1) was incorporated in the ND virosomes. The engineered virosomes were efficiently fused with Vero cells, and GFP was expressed in the transfected cells, confirmed by fluorescent microscopy. It indicated the presence of intact HN and Fusion viral envelop glycoproteins on ND virosomes and its ability to fuse animal cells. Previously similar experiments were conducted to evaluate the fusogenic attributes of ND virosomes [34, 36].

Following a detailed investigation for the characterization of NDV strain Okara, virosome production was done at a mass scale for the formulation of indigenous ND virosome. Briefly, sucrose-purified ND virosome was resuspended in phosphate-buffered saline (PBS), pH 7.2, at a protein concentration of 2 mg/ml [14, 36]. To ensure vaccine inactivation, reconstituted virosomes (diluted 1 : 10 in PBS) were tested by inoculation into 9-to-11-day-old SPF chicken embryos as above and monitored for mortality [14]. To ensure vaccine sterility, it was inoculated on different culture media for bacterial and fungal contamination. There was no turbidity in the broth, or no growth observed on any agar media. No bacteria including mycoplasma and fungal contamination were observed [23]. The safety of the test vaccine was confirmed by embryo inoculation, and there were no lesions observed in chicken embryos even up to 7 days postinoculation of virosome [23]. Moreover, the stability of the ND virosome vaccine was assessed by dynamic light scattering (DLS) and found that the vaccine was stable on storage at 4°C, 25°C, and 37°C for different periods of time [23].

*In vivo* trials in experimental chicken indicated that the HI antibody titers were protective and the highest in G2 vaccinated with a live vaccine, followed by virosome (G1) and killed (G3) vaccines, respectively. The GMTs were very low and nonsignificant (*p* > 0.05) in all groups before vaccination, whereas a significant difference (*p* < 0.05) in GMTs was observed in all vaccinated groups from the negative control group (G4) throughout the experiment. The antibody titers were maximum in the virosome vaccine group (G1) with the highest GMTs as 83.18 and 77.62 at 21^st^ day and 28^th^-day postvaccination, respectively. Likewise, titers were also found maximum in the case of the live vaccine group (G2) with GMTs values as 89.13 and 77.62 at 21^st^ day and 28^th^-day postvaccination, respectively. A similar trend was also observed for the killed vaccine (G3) with nonsignificant (*p* > 0.05) differences in GMTs as compared to virosome and live ND vaccines. The findings of the experimental trial are comparable to the findings [14, 34, 36].

A challenge protection assay was done and upon challenge with wild NDV strain, virosome-based test vaccine showed 100% protection, whereas commercially available live vaccine (La Sota) and killed vaccines exhibited 90% and 80% protection, respectively. A study reported 70% to 90% protection by the virosome vaccine against challenge with virulent virus [36], whereas other studies reported 100% protection following challenge [14]. A recent study reported that VLPs alone and in combination with alum impart sufficient protection following challenge [34].

Based on the overall results of the present study, it was concluded that the virosome vaccine prepared from an indigenous virulent strain of NDV was found to be immunogenic and exhibited good clinical protection against challenge in broiler chicken. We recommended that the prepared vaccine needs further studies to evaluate its effects on cell-mediated and mucosal immunity, its efficacy in immunization of backyard/rural poultry, and commercial poultry against ND.

## Figures and Tables

**Figure 1:** Ethidium bromide stained 1% agarose gel representing the PCR amplified F gene of indigenous NDV approximately 800 bp (Lane 1). Complete map of ladder shown at left side of image (M: marker; lane 1: virus; lane 2: negative control).

**Figure 2:** Sequences were obtained from GenBank and dendrogram was constructed by neighbor-joining method, the scale represents evolutionary distance overtime. The tree represents City or Province, Country name, and GenBank accession number.

**Figure 3:** Coomassie brilliant blue-stained 8% acrylamide gel represents five different proteins of indigenous ND virus. M: protein marker and lane 1: viral proteins (HN: viral hemagglutinin-neuraminidase; F: fusion; N: nucleocapsid; PH: phospho; M: matrix proteins).

**Figure 4:** Transmission electron micrograph displaying the structural morphology of ND virosome: oval to spherical in shape with 75 to 200 nm in size.

**Figure 5:** Acrylamide gel representing the comparison of ND virosomes and whole virus proteins (M: marker; lane 1&2: virosomal proteins; and 3: viral proteins).

**Figure 6:** Ethidium bromide-stained 1% agarose gel representing the nested PCR amplified plasmids portion lying between CMV and SV40 region (900 bp). Complete map of ladder shown at left side of image (M: marker; lane 1 to 4: amplified plasmid; and lane 5: negative control).

**Figure 7:** Transfection experiments confirmed the ability of ND virosomes to bind the animal cells. Cells were firstly examined under bright field (A: control untransfected cells and B: transfected cells), then observed under green fluorescent filter mode (C: control untransfected cells; and D: transfected cells).

**Table 1:** The HI antibody titers at 21st day postvaccination.

	HI antibody titers			
No. of birds	G1	G2	G3	G4
1	32	32	128	0
2	128	128	256	2
3	256	64	128	0
4	128	256	128	0
5	64	64	32	2
6	64	32	32	0
7	32	64	64	0
8	128	256	128	2
9	128	128	32	2
10	64	128	128	0
GMT	83.18^a^	89.13^a^	83.18^a^	1.31^c^

(*p* < 0.05).

**Table 2:** The HI antibody titers at 28th day postvaccination.

	HI antibody titers			
No. of birds	G1	G2	G3	G4
1	64	32	128	0
2	64	64	64	0
3	128	64	32	2
4	256	256	256	0
5	64	32	64	0
6	32	64	32	0
7	64	32	64	2
8	128	128	128	0
9	128	256	64	0
10	32	128	32	0
GMT	77.62^a^	77.62^a^	67.60^a^	1.14^c^

(*p* < 0.05).

**Table 3:** Morbidity and mortality in broiler chicks up to 10 days postchallenge with different ND vaccines.

Groups	Vaccine	No. of birds challenged	No. of diseased birds	Morbidity %	No. of birds died	Mortality rate	Protection rate
G1	Virosome	10	1	10	0	10	100
G2	La Sota	10	2	20	1	0	90
G3	Killed	10	3	30	2	20	80
G4	Nonvaccinated control	10	10	100	9	90	10

## Data Availability

The data that support the findings of this study is included in the manuscript.
